The article "Protective Effects of Herba Houttuyniae Aqueous Extract against OVA-Induced Airway Hyperresponsiveness and Inflammation in Asthmatic Mice" was published in 2022. Journal: Evid Based Complement Alternat Med.

# Protective Effects of *Herba Houttuyniae* Aqueous Extract against OVA-Induced Airway Hyperresponsiveness and Inflammation in Asthmatic Mice

**DOI:** 10.1155/2022/7609785

**Published:** 2022-11-11

**Authors:** Yu Yang, Qingzhong Lai, Chenyu Wang, Gaoli Zhou

**Affiliations:** ^1^Medical Laboratory, Fuyang District Maternal and Child Health Hospital, Hangzhou 311400, China; ^2^Department of Chinese Medical Massage, Zhejiang Integrated Traditional and Western Medicine Hospital, Hangzhou 310003, China; ^3^Pediatric Department, Fuyang District Maternal and Child Health Hospital, Hangzhou 311400, China

## Abstract

*Herba Houttuyniae* is the well-knownfood-medicine herb with the special taste and smell. It is also widely used in south China for prevention of various chronic pulmonary inflammatory diseases including asthma. However, the active ingredients and therapeutic mechanism of this herb remain obscure. In this study, network pharmacology technology was employed to investigate the effects of *Herba Houttuyniae* aqueous extract (HHAE) on OVA-induced airway hyperresponsiveness and inflammation. The results showed that six compounds (isoramanone, kaempferol, 1-methyl-2-nonacosyl-4-quinolone, C09747, spinasterol, and quercetin) were found to be mainly responsible for the therapeutic effects of the herb, which totally regulated the expressions of 168 asthma-related proteins. All those targets involved in the signal transduction of the prolactin signaling pathway, central carbon metabolism in cancer, EGFR tyrosine kinase inhibitor resistance, endocrine resistance, and VEGF signaling pathway. The in vivo experiment also revealed that orally administrated with HHAE alleviated airway hyperresponsiveness and inflammation in OVA-induced asthmatic mice. It significantly decreased the counts of neutrophils, eosinophils, and lymphocytes as well as the levels of IL-1*β*, IL-4, IL-6, and IL-13 in BALF of asthmatic mice. Mechanically, HHAE downregulated both the mRNA and protein expressions of p38 MAPK, PI3K, AKT, and VEGF in the lung tissues of asthmatic mice. Therefore, HHAE improved OVA-induced airway hyperresponsiveness and inflammation in mice and could be a potential supplement for asthma treatment.

## 1. Introduction

Asthma is a chronic inflammatory disease of the airways, commonly seen in people with allergies. Its clinical symptoms, such as breathlessness, chest tightness, and breath shortness, are occurring mostly at night or early in the morning. According to statistics, there are more than 300 million of asthma sufferers worldwide, and an estimated 30 million in China [1, 2]. The recent treatment of asthma in the clinic is mainly based on asthma calming, anti-inflammatory, and bronchodilatation, by using glucocorticoids, leukotriene receptor antagonists, and beta2-agonists, but long-term use of those agents will lead to a decrease in the patient's immunity but an increase in drug resistance [3–5].

Asthma belongs to the category of “pant” and “croup” in Traditional Chinese medicine. In the theory of traditional Chinese Medicine (TCM), the main pathogenesis of asthma is the internal accumulation of phlegm in the lungs, combined with external influences, diet, emotions, and fatigue [6]. TCM has accumulated rich experiences in treating asthma, and especially it can improve the compliance of patients in remission stage and early stage [7, 8]. Many TCMs, such as Xiaoqinglong decoction, Perilla, Pinellia ternata, Armeniacae Semen, and Eriobotrya japonica, presented better curative effects than glucocorticoids [9–14]. *Herba Houttuyniae* is the dried root of the plant Houttuynia cordata Thunb., which belongs to the family *Saururaceae*. It has been widely used as the antiasthmatic and cough medicine for various respiratory diseases for years [15]. Due to its special taste and smell, especially popular in the summer, this plant is sliced and served like a salad with various dressings [16]. Previous studies had demonstrated its obvious protective effects against various stimuli-induced lung discords, including influenza infection, chronic obstructive pulmonary disease, and even COVID-19 via mediating TLR4 activation, reducing oxidant stress, and directly inhibiting viral encode RNA-dependent RNA polymerase [17–21]. In addition, this herb exerted obvious immunomodulation through enhancing the phagocytic activity of the neutrophils and promoting lymphocyte proliferation [22], but the long-term treatment with herbal ethanol extract with the doses less than 250 mg/kg/day (equal to its clinical dosage) did not have significant hepatotoxicity and nephrotoxicity in rats [23]. However, the active ingredients and therapeutic mechanisms of this herb are not clear. In this paper, we investigated the active ingredients, potential targets, and signaling pathways for the treatment of asthma based on network pharmacology, and then experimentally validated the antiasthmatic mechanism of this herb in mice, to provide theoretical basis for future clinical use.

## 2. Materials and Methods

### 2.1. Herbal Extracts and Reagents

The herb was obtained from the Huadong Medicine Co. Ltd, China, and identified by Prof. Qingzhong Lai, Zhejiang Integrated Traditional and Western Medicine Hospital, Hangzhou, China. One kilogram of the dry herb was soaked in 10 L of water for 30 min and then heated for 1 h. After being filtered, the supernatant was concentrated to 500 ml and then centrifuged at 2000 rpm for 20 min to remove the impurity. All the chemical reagents were obtained from Sinopharm Co. Ltd., Shanghai, China.

### 2.2. HPLC Analysis

About 20 ml of 80% methanol solution, 0.5 ml of 1% (V/V) hydrochloric acid solution, and 1 ml of aqueous extract were added into the round-bottomed flask, and then reflux hydrolyzed at 85°C for 1 h. After filtration by filter paper, the extracts were fixed with methanol to 50 ml, shook well, and filtered through a 0.45 *μ*m membrane before use.

The quality control of the herbal extract [i.e., *Herba Houttuyniae* aqueous extract (HHAE)] was carried out on an Agilent 1260 LC system. The Agilent Eclipse plus C_18_ column (100 mm × 4.6 mm, 5 *μ*m) was used and the mobile phase consisted of methanol and 0.4% phosphoric acid solution (45 : 55, V/V) with the current speed at 0.8 ml/min. The detection wavelength and the column temperature were set at 360 nm and 30°C, respectively.

### 2.3. Target Screening of the Active Ingredients in *Herba Houttuyniae*

Using “houttuynia (or yuxingcao)” as the key word, we employed the TCMSP database (https://tcmspw.com/tcmsp.Php) and the TCMID database (https://www.megabionet.org/tcmid/) to retrieve the main chemical compounds in *Herba Houttuyniae*. But only the compounds, which had the oral bioavailability (OB) ≥30%, drug-likeness (DL) ≥0.18, and drug half-life (HL) ≥4 h, were considered as the eligible active compounds in *Herba Houttuyniae*. After the Canonical SMILES of each candidate compound in the PubChem database was obtained(https://pubchem.ncbi.nlm.nih.gov/), SwissTargetPrediction online service (https://www.swisstargetprediction.ch/) was used to find the potential target s of those 6 compounds. The keyword “asthma” was used in the GeneGards database to gain the well-known target set related to asthma, and then Venny web-software (https://bioinfogp.cnb.csic.es/tools/venny/index.htmL) was used to select common targets of *Herba Houttuyniae* for the treatment of asthma. Finally, the String database (https://string-db.org/) was used to obtain the protein–protein interaction and KEGG enrichment.

### 2.4. Asthmatic Model and HHAE Treatment

A total of 60 male Balb/c mice were randomly divided into 6 groups: normal control group, asthma model group, positive control group [dexamethasone (DEX), 10 mg/kg], and HHAE-treated groups (400, 200, and 100 mg/kg, respectively). All groups were sensitized by intraperitoneal injection of 0.1 ml/10 g of sensitizing solution, except for the normal control group, which was injected intraperitoneally with 0.1 ml/10 g of saline at day 1 and day 14, respectively. From day 22 onwards, the drugs were administered to each group of mice 24 h before each nebulization, while the normal control group and the asthma model group were given saline. The mice were anesthetized with ether 24 h after the last nebulization. The tissues of the left lung were prepared and stained by HE. The pathology scores were analyzed by two independent physicians as previous reports [24–26].

### 2.5. Detection of Airway Hyperresponsiveness

After 48 h of the last OVA booster, awake mice were placed on a lung function system and the mean baseline readings were recorded over 3 min, and nebulized with acetylcholine (2.5–50.0 g/L) for 3 min. The enhanced pause (Penh) was calculated according to the instructions for the detection of airway hyperresponsiveness to reflect the degree of increased airway responsiveness.

### 2.6. Cell Count in Bronchoalveolar Lavage Fluid (BALF)

The mouse was anesthetized with ether and fixed on a mouse plate. The lung tissue was quickly separated, the right main bronchus was ligated, 1 ml of saline was injected from the left main bronchus, and the alveolar lavage fluid was repeatedly withdrawn after about 1 min (recovery rate>80%). After being centrifuged at 3000 rpm for 15 min, the precipitate was resuspended with 0.5 ml of saline. The number of leukocytes was counted by using automated blood cells counter (Sh-taiyi biotech Company, China).

### 2.7. RT-PCR Detection

About 40 mg of mouse lung tissues was ground in a mortar, pestle with an appropriate amount of liquid nitrogen, and then mixed with 1 ml of RNA extraction reagent for lysis and digestion according to the kit instructions (Beyotime Biotechnology Co., China). The sequences of the primers were used in this study as follows: p38 MAPK: forward primer 5′-TAGTTACCTTGCCACTTTGGCT-3′, reverse primer 5′-TGCACCAT GGCCTTCCTAAA-3′, product length 346 bp; PI3K: forward primer 5′-CTCCGTGCAGGGACAAAGAG-3′, reverse primer 5′-CCTCCGAACAGACTG CATCA-3′, product length 292 bp; Akt: forward primer 5′-GTTTTGTTTCTCGGATGCGCT-3′, reverse primer 5′-CATGGTCGCGTCAGTCCTTA-3′, product length 223 bp; VEGF Forward primer 5′-TTTGCCAAGGGTCCTCACAC-3′, reverse primer 5′-AAGTAAACTGCATGCTGGGC-3′, product length 168 bp; *β*-actin forward primer 5′-TTACAGGAAGTCCCTCACCC-3′, reverse primer 5′-ACACAGAAGCAA TGCTGTCAC-3′, product length 110 bp.

### 2.8. Western Blot Analysis

The expressions of the testing proteins in mouse lung tissues were measured by western blot analysis. Protein extraction kits (Beyotime, Shanghai, China) were used to extract total protein from mouse lung tissues; protein concentrations were determined by BCA method. SDS-PAGE was performed, and then membranes were transferred and closed. The antibodies (1 : 2000; Proteintech, USA) were incubated overnight at 4°C, and antirabbit IgG (1 : 5000; Proteintech, USA) was added and incubated for 1 h at room temperature, protected from light. Enhanced chemistry was developed and the protein bands were analyzed in gray scale using ImageJ software.

### 2.9. Flow Cytometry for the Detection of Th1 and Th2 Levels

Flow cytometry was performed to detect the levels of IFN-*γ* and IL-4 in CD4^+^ T lymphocytes, respectively. Under aseptic conditions, the spleen was isolated from the back of the mouse, and then soaked in the 1640 complete medium. After being completely grounded, the lymphocyte separation medium was added and centrifuged with 3 000 r/min for 30 min at room temperature. The middle turbid cell layer was collected and washed once by a 1640 complete medium. The cells were resuspended, counted by a cell counter at the concentration of 1 × 10^8^ cells/ml, distributed into a 12-well plate, and mixed with cell stimulant. After incubation in the incubator (Subo Co. Ltd., Suzhou, China) for 16 h, 100 *μ*l of cell suspension was added to the flow tube, mixed with antimouse CD4^+^ APC and incubated at 4°C for 30 min. The cells were centrifuged at 1400 r/min for 5 min. IC fixation was added, incubated at room temperature for 20 min, washed by PBS, and incubated with fixation/permeabilization at 4°C for 20 min in dark. Finally, the cells were incubated with antimouse-IL-4-PE, and antimouse-IFN-*γ*-FITC for 30 min at 4°C. After being centrifuged at 1400 r/min for 5 min and washed by PBS, the cells were resuspended in buffer and analyzed by flow cytometry (Beckman, USA).

### 2.10. Statistical Analysis

Data were analyzed statistically by using Graphpad Prism 8.0, and showed as means ± SD. One-way ANOVA was used for multiple group comparisons. *P* < 0.05 indicated a statistically significant difference between the two groups.

## 3. Results

### 3.1. The Active Compounds in *Herba Houttuyniae*

Fifty chemical compounds were obtained from the TCMSP database when we used the keyword “yuxingcao” for search. After filtered by setting “OB>30%, DL > 0.18, and HL 4 h,” only 6 compounds (isoramanone, kaempferol, 1-methyl-2-nonacosyl-4-quinolone, C09747, spinasterol, and quercetin) were collected, as shown in Table 1. To control the quality of the herbal extract, the contents of kaempferol and quercetin in HHAE were detected by HPLC method. As shown in Figure 1, both kaempferol and quercetin could be detected in HHAE, and their contents were 38.4 mg/g and 12.6 mg/g, respectively.

Further target prediction by using SwissTargetPrediction showed that those 6 compounds could target 248 proteins. Among them, 168 common targets were considered as candidate targets of *Herba Houttuyniae* for the treatment of asthma, which were also found to be closely related to the development of asthma (Figure 2(a)).

Furthermore, interaction among the 168 candidate targets were constructed by the STRING web-service, and confidence score 0.7 was set as a qualification condition. As shown in Figure 2(b), the interaction network of the 168 candidate targets was drawn. Network stats was presented as follows: number of nodes was 298, number of edges 1087, average node degree 7.3, average local clustering coefficient 0.461, and PPI enrichment *P* value was less than 0.001. The top 10 highest degree of targets were EGFR, JAK1/2, MAPK14, VEGF, SRC, mTOR, PI3K, and GSK3B, which might be the critical targets of HHAE for the treatment of asthma (Figure 2(c)). More notably, the KEGG enrichment results also revealed that the regulation of prolactin signaling pathway, pathways in cancer, endocrine resistance, EGFR tyrosine kinase inhibitor resistance, proteoglycans in cancer, central carbon metabolism in cancer, ErbB signaling pathway, insulin resistance, and cAMP signaling pathway contributed to the therapeutic effects of HHAE against OVA-induced asthma (Figure 3).

### 3.2. HHAE Reduced Airway Responsiveness in OVA-Induced Asthmatic Mice

When the dose of methacholine was increased to 10–50 g/L, the airway responsiveness of mice in the OVA group was significantly increased. There were significant differences in Penh values between the model group and the normal control group (*P* < 0.05), indicating the increased airway responsiveness after OVA challenge. Compared with the OVA group, the Penh values of mice in DEX- and HHAE-treated groups were significantly lower than that of mice in model group (*P* < 0.05). Notably, when exposed with 50 g/L of methacholine, there were no significant differences in Penh values between the DEX-treated group and 400 mg/kg HHAE-treated group (*P* < 0.05), indicating the remarkable inhibition of HHAE on OVA-induced airway responsiveness in asthmatic mice.

### 3.3. HHAE Reduced Lung Inflammation in OVA-Induced Asthmatic Mice

After OVA sensitization, the tissues of the mouse lung presented obvious inflammatory cell infiltration with the increased pathology scores in Figure 4(a), while treatment with DEX and HHAE could ameliorate the inflammatory response and significantly reduce the pathology scores compared with the model group (*P* < 0.05). Compared with the normal control group, the number of neutrophils, lymphocytes, and eosinophils in BALF of asthmatic mice were significantly increased (*P* < 0.05). Compared with the asthma model group, the counts of those inflammatory cells in BALF in the HHAE-treated groups were significantly reduced (Figure 4(b)). Furthermore, the levels of proinflammatory cytokines in BALF were closely consistent with the trends of inflammatory cells in BALF. Compared with the normal control group, the levels of IL-1*β*, IL-4, IL-6, and IL-13 in BALF of asthmatic mice were much higher than those in normal control mice (*P* < 0.05). Treatment with HHAE (100–400 mg/kg) decreased the levels of those cytokines in BALF dose-dependently (Figure 5). Similarly, the proportion of Th1 cells was markedly decreased in the spleens of asthmatic animals compared with that in the control group (*P* < 0.05), while the proportion of Th1 cells was sharply enhanced; however, HHAE treatment reversed those trends. Those results indicated that HHAE reduced lung inflammation in OVA-induced asthmatic mice.

### 3.4. HHAE Inhibited the Activation of PI3K/AKT and VEGF Pathways in OVA-Induced Asthmatic Mice

The results in Figures 6 and 7 displayed that the mRNA and protein expressions of p38 MAPK, PI3K, Akt, and VEGF in the lung tissues of normal mice were very low. However, after repeated sensitization of OVA, the expressions of those markers in the lung tissues of asthmatic mice were significantly upregulated. Oral administration with HHAE (100–400 mg/kg) could significantly decrease the mRNA and proteins expressions of p38 MAPK, PI3K, Akt, and VEGF.

## 4. Discussion

Asthma is a common disease of the respiratory system characterized by chronic inflammation, airway hypersensitivity, and remodeling due to the involvement of various inflammatory mediators, cytokines, and signaling molecules. Infiltration of lung tissue by inflammatory cells such as eosinophils, neutrophils, and lymphocytes has been found to be the main cause of airway inflammation and asthma allergy [27]. The activation of eosinophils induces apoptosis of alveolar and airway epithelial cells by releasing large amounts of basic proteins, leukotrienes, and free radicals, causing structural remodeling and hypersensitivity of airways [28]. During the inflammatory response, eosinophils also induce lymphocytes to synthesize and release cytokines such as IL-1*β*, IL-4, IL-6, and IL-13, which promote and exacerbate asthma attacks. Neutrophils can accumulate in the airways and alveoli and release chemokines that promote and exacerbate inflammatory responses, leading to asthma attacks and exacerbations [29]. In addition, CD3^+^, CD4^+^, and CD8^+^ T cells are the main subtypes of the primary T cells. Previous studies had demonstrated that Th1/Th2 imbalance contributed to the development of allergic asthma; Th1 cells are mainly involved in cellular immune responses, while Th2 cells can induce specific humoral immunity. When the Th1/Th2 ratio is in dynamic equilibrium in the body, the immune system is in relative balance [30–33]. OVA challenge disrupted the balance to some extent; however, the imbalance could be partially reversed by HHAE treatment. Therefore, inhibiting and reducing the inflammatory response and inflammatory cell infiltration in the lungs of asthma patients is the main strategy to prevent and relieve asthma attacks. Natural products exhibit the complex chemical backbone and the rich functionalization, making them unique biological activity and unique properties that cannot be replaced as lead compounds in pharmaceutical research [34–37]. Many antiasthmatic drugs derived from the herbal medicine, such as ephedrine and glycyrrhizic acid, have been used widely in the clinic for prevention and treatment of airway inflammation and asthma [38–41]. Given the diversity of the compounds in the plant extract, network pharmacology technology was employed to find the potential active compounds in HHAE which may be responsible for its therapeutic effects against OVA-induced asthma. Total six compounds (isoramanone, kaempferol, 1-methyl-2-nonacosyl-4-quinolone, C09747, spinasterol, and quercetin) were obtained by network pharmacology analysis and the contents of kaempferol and quercetin were determined by HPLC method to prove the reliability of network pharmacology analysis. Further analysis showed that those bioactive compounds could totally regulate the expressions of 168 asthma-related proteins. Then, the results of animal experiments also demonstrated that HHAE significantly reduced the neutrophil, lymphocyte, and eosinophil counts in alveolar lavage fluid of asthmatic mice, and it also significantly improved the histopathological changes of lung tissues in mice with asthma, resulting in a significant reduction of airway remodeling and alveolar damage in mice with asthma.

Studies have reported that the p38 MAPK/PI3K signaling is one of the important signaling pathways mediating the inflammatory response in asthma [42, 43]. p38 MAPK is an important signaling regulatory molecule that is activated to transmit free radicals, inflammatory stimuli, and other damaging signals to cells [44]. Activation of p38 MAPK activates the PI3K/Akt signaling pathway by phosphorylating p38 MAPK, which further activates the PI3K/Akt signaling pathway [45]. p38 MAPK/Akt activation activates factors such as VEGF, which promotes the proliferation of airway structural cells, including alveolar epithelial cells, bronchial endothelial cells, fibroblasts/myofibroblasts, and bronchial smooth muscle cells, can contribute to inflammation and angiogenesis in various pulmonary inflammatory diseases, making the lumen narrower and participating in airway remodeling [46, 47]. Moreover, VEGF accelerated M2 macrophage infiltration and disrupted the airway epithelial barrier in lung tissues of asthmatic animals [48–51]. Emerging evidence also displayed that VEGF has associations with thromboembolism and tissue injury/repair in COVID-19 and viral infection, indicating the promotion of secondary airway inflammation [52–54]. The results of this study showed that HHAE significantly reduced the expression levels of p38 MAPK, PI3K, Akt, and VEGF mRNA and protein in lung tissue of asthmatic mice, suggesting that the mechanism of HHAE alleviating asthma inflammation is related to the inhibition of the p38 MAPK/PI3K signaling pathway.

In summary, HHAE mainly contained flavonoids and obviously improved airway hyperresponsiveness and inflammation in OVA-induced asthmatic mice via inactivation of MAPK/PI3K/AKT/VEGF pathways. Therefore, it could be used as a supplement for treatment and prevention of allergic asthma.

## Figures and Tables

**Figure 1:** HPLC chromatograms of chemical standards and HHAE samples. (a) the chromatogram of the chemical standards (1. Quercetin; 2. kaempferol). (b) the chromatogram of the herbal samples.

**Figure 2:** The target profiles of 6 active compounds in HHAE on OVA-induced asthma. (a) Venn diagrams showed the overlap between asthma-related genes derived from GeneCards and HHAE targets predicted by SwissTargetPrediction Server. (b) Network interactions among 168 overlapped targets of HHAE. The edges indicate both functional and physical protein associations; line thickness indicates the strength of data support. (c) Network correlation of the Top 10 genes.

**Figure 3:** Identification and enrichment analysis of 168 targets of 6 active compounds in HHAE. The diagram showed the top 10 pathways enriched by 168 functional protein associations.

**Figure 4:** Effects of HHAE on inflammatory response in asthmatic mice. (a) HHAE decreased the pathology scores of asthmatic mice. (b) HHAE reduced the infiltration of inflammatory cells in BALF of asthmatic mice. Data were showed as mean ± SD. Different letters indicated statistically significant differences, *P* < 0.05.

**Figure 5:** Effects of HHAE on the levels of proinflammatory cytokines in BALF and splenocytes of asthmatic mice. (a) HHAE reduced the levels of IL-1*β*, IL-4, IL-6, and IL-13 in BALF of asthmatic mice. (b) HHAE restored the balance of Th1/Th2 cells in the spleens of asthmatic mice. Data were showed as mean ± SD. Different letters indicated statistically significant differences, *P* < 0.05.

**Figure 6:** The changes of airway hyperresponsiveness in OVA-induced asthmatic mice. Data were showed as mean ± SD. Different letters indicated statistically significant differences, *P* < 0.05.

**Figure 7:** Effects of HHAE (100–400 mg/kg) on expressions of PI3K, Akt, p38 MAPK, and VEGF mRNAs as well as proteins in the lung tissues of OVA-induced asthmatic mice. Data were showed as mean ± SD. Different letters indicated statistically significant differences, *P* < 0.05.

**Table 1:** The ADME parameters of 6 active compounds in *Herba Houttuyniae*.

No.	Name	MW	OB (%)	DL	HL
1	Isoramanone	39.97	39.97	0.51	4.79
2	Kaempferol	41.88	41.88	0.24	14.74
3	1-methyl-2-nonacosyl-4-quinolone	31.54	31.54	0.50	16.13
4	Ruvoside_qt	36.12	36.12	0.76	7.21
5	Spinasterol	42.98	42.98	0.76	5.32
6	Quercetin	46.43	46.43	0.28	14.40

ADME, absorption, distribution, metabolism, and excretion; MW, molecular weight; OB, oral bioavailability; DL, drug likeness; HL, Drug half-life.

## Data Availability

The data used to support the findings of this study are available from the corresponding author upon request.
